The article "Metformin Protects From Rotenone–Induced Nigrostriatal Neuronal Death in Adult Mice by Activating AMPK-FOXO3 Signaling and Mitigation of Angiogenesis" was retracted in 2026. Reasons: duplicated images; overlap with earlier publications; unreliable data; unreliable results or conclusions.

# Metformin Protects From Rotenone–Induced Nigrostriatal Neuronal Death in Adult Mice by Activating AMPK-FOXO3 Signaling and Mitigation of Angiogenesis

**DOI:** 10.3389/fnmol.2020.00084

**Published:** 2020-06-18

**Authors:** Sabah H. El-Ghaiesh, Hoda I. Bahr, Afaf T. Ibrahiem, Doaa Ghorab, Suliman Y. Alomar, Noha E. Farag, Sawsan A. Zaitone

**Affiliations:** ^1^Department of Pharmacology, Faculty of Medicine, University of Tabuk, Tabuk, Saudi Arabia; ^2^Department of Pharmacology, Faculty of Medicine, Tanta University, Tanta, Egypt; ^3^Department of Biochemistry, Faculty of Veterinary Medicine, Suez Canal University, Ismailia, Egypt; ^4^Department of Pathology, Faculty of Medicine, Mansoura University, Mansoura, Egypt; ^5^Doping Research Chair, Department of Zoology, College of Science, King Saud University, Riyadh, Saudi Arabia; ^6^Department of Physiology, Faculty of Medicine, Suez Canal University, Ismailia, Egypt; ^7^Department of Physiology, College of Medicine, Taif University, Taif, Saudi Arabia; ^8^Department of Pharmacology and Toxicology, Faculty of Pharmacy, Suez Canal University, Ismailia, Egypt; ^9^Department of Pharmacology and Toxicology, Faculty of Pharmacy, University of Tabuk, Tabuk, Saudi Arabia

**Keywords:** AMPK-FOXO3, cleaved caspase 3, metformin, oxidative stress, rotenone-induced parkinsonism, vascular endothelial growth factor

## Abstract

Parkinson’s disease (PD) is a neurodegenerative disease that affects substantia nigra dopamine neurons. Many studies have documented the role of oxidative stress and angiogenesis in the pathogenesis of PD. Metformin (MTF) is an antidiabetic medication and AMP-activated protein kinase (AMPK) regulator that has shown antioxidant and antiangiogenic properties in many disorders. The aim of this study is to investigate the neuroprotective effect of MTF in a mouse model of rotenone-prompted PD with a highlight on its influence on the AMPK/forkhead box transcription factor O3 (FOXO3) pathway and striatal angiogenesis. In the running study, PD was induced in mice using repeated doses of rotenone and concomitantly treated with MTF 100 or 200 mg/kg/day for 18 days. Rotarod and pole tests were used to examine the animals’ motor functionality. After that, animals were sacrificed, and brains were isolated and processed for immunohistochemical investigations or biochemical analyses. Oxidant stress and angiogenic markers were measured, including reduced glutathione, malondialdehyde, the nuclear factor erythroid 2–related factor 2 (Nrf2), hemoxygenase-1, thioredoxin, AMPK, FOXO3, and vascular endothelial growth factor (VEGF). Results indicated that MTF improved animals’ motor function, improved striatal glutathione, Nrf2, hemoxygenase-1, and thioredoxin. Furthermore, MTF upregulated AMPK-FOXO3 proteins and reduced VEGF and cleaved caspase 3. MTF also increased the number of tyrosine hydroxylase (TH)–stained neurons in the substantia nigra neurons and in striatal neuronal terminals. This study is the first to highlight that the neuroprotective role of MTF is mediated through activation of AMPK-FOXO3 signaling and inhibition of the proangiogenic factor, VEGF. Further studies are warranted to confirm this mechanism in other models of PD and neurodegenerative diseases.

## Introduction

Rotenone is a plant-extracted chemical with a wide application in pesticides and insecticides. Rotenone is classified by WHO as class-II pesticide with a moderate hazards (World Health Organization and International Programme on Chemical Safety, 2010). Rotenone is proofed to produce a validated experimental model of Parkinson’s disease (PD) referring to suppression of complex I and activation of microglia properties resulting in oxidative stress, inflammatory response, neurotoxicity, and locomotor and behavioral alterations (Drolet et al., 2009; Xiong et al., 2012; Johnson and Bobrovskaya, 2015). PD is characterized by high mitochondrial reactive oxygen species (ROS) production with resultant DNA deletions, degeneration of dopaminergic neurons within substantia nigra pars compacta (SNpc) favoring cell death, and impaired autophagy (Button et al., 2015; Ordonez et al., 2018). Angiogenesis plays an important role in the pathogenesis of PD as has been reported in clinical and animal studies (Faucheux et al., 1999; Barcia et al., 2005; Janelidze et al., 2015).

Metformin (MTF) is a commonly used antidiabetic drug due to its hypoglycemic, antioxidant, and anti-inflammatory effsect (Mahmood et al., 2013; Wang et al., 2016). There is growing evidence for the benefit of metformin to counteract age-related diseases, such as neurodegenerative diseases (Rotermund et al., 2018). One clinical study revealed that MTF decreased incidence of PD in a type-2 diabetic patient (Wahlqvist et al., 2012). Recently, some studies have highlighted the neuroprotective properties of MTF and its ability to decrease risk of PD both *in vitro* and *in vivo*. MTF prevents primary cortical neuron apoptosis *in vitro* by delayed permeability transition pore opening (El-Mir et al., 2008). MTF was reported to increase Bcl-2, decrease Bax expression, and reduce activation of caspase-9 and caspase-3 in ethanol-mediated apoptosis in prenatal rat cortical neurons (Ullah et al., 2012). *In vivo*, oral administration of MTF in 1-methyl-4-phenyl tetrahydropyridine (MPTP)-treated mice improves locomotor activities and antioxidant status and amends neurogenesis (Patil et al., 2014). Similarly, MTF protects against cytotoxicity and redox imbalance initiated by rotenone in rat erythrocytes (Tripathi et al., 2019).

Many researches pronounced that MTF activates AMP-activated protein kinase (AMPK)- mediated neuronal autophagy and anti-apoptosis. For instance, chronic MTF was reported to protect from stroke via AMPK activation (Li et al., 2010). Further, MTF enhances brain AMPK with induction of autophagy in a model of middle cerebral artery occlusion (Jiang et al., 2014) and improvement of motor impairment in MPTP parkinsonian mice (Lu et al., 2016). Moreover, MTF ameliorates SN gliosis in experimental parkinsonism (Bayliss et al., 2016) and spinal cord injury via increasing Beclin-1, BCl2, and LC3B-II expression and decreased phosphorylation of the mammalian target of rapamycin (mTOR), nuclear factor-κB (NF-κB) expression, and caspase 3 activation (Wang et al., 2016).

Forkhead box transcription factor O3 (FOXO3) is an important determinant of dopaminergic neuronal survival through differing oxidant stress and macroautophagic mechanisms (Pino et al., 2014; Curry et al., 2018). Recently, MTF has been shown to upregulate erythroid FOXO3 and improve hemoglobinopathy (Zhang Y. et al., 2018). Additionally, MTF was reported to enhance cellular redox homeostasis through the AMPK-mediated FOXO3 pathway (Hou et al., 2010). MTF plays an important antiangiogenic role as has been demonstrated in *in vivo* and *in vitro* studies on cancer (Falah et al., 2017; Qian et al., 2018; Zhang H.H. et al., 2018; Moschetta et al., 2019), diabetic retinopathy (Han et al., 2018), and cerebral stroke (Jin et al., 2014).

The influence of MTF on the AMPK/FOXO3 pathway and striatal angiogenesis has not been examined in PD. The running work aimed at exploring the AMPK/FOXO3 activating and antioxidant role of MTF in rotenone-parkinsonian mice and the ability of MTF to mitigate angiogenesis. The work involved checking of the motor function and assessment of the integrity of SNpc neurons.

## Materials and Methods

### Animals and Ethics Approval

In this study, adult male Swiss albino mice (21–30 g in weight, 8–10 weeks in age) were used. Mice were purchased from the M. Rashed Company for experimental animals and kept under clean laboratory settings and a normal light–dark cycle. Water and food were allowed *ad libitum*. Male Swiss albino mice were selected as they have been frequently used in previous models of parkinsonism (Zaitone et al., 2019). Experimental protocols and animal handling procedures were officially approved by the research ethics committee (approval number 201608RA4), Faculty of Pharmacy, Suez Canal University, in compliance with the National Institute of Health Guide for the Care and Use of Laboratory Animals (NIH Publication No. 8023, revised 1978).

### Chemicals and Drugs

Rotenone (Sigma-Aldrich, St. Louis, MO, United States) was dissolved in commercial-grade sunflower oil. Metformin HCl was a gift from Medical Union Pharmaceuticals (Ismailia, Egypt) and was dissolved in distilled water.

### Experimental Model and Study Groups

Animals (*n* = 36) were equally and randomly divided into six groups, each consisting of six animals.

*Group 1 (vehicle):* Mice received nine subcutaneous (s.c.) injections of the vehicle (sunflower oil, 4 ml/kg) every 48 h.

*Group 2 (rotenone):* Parkinsonism was induced by injecting nine doses of rotenone (1 mg/kg, s.c.), every 48 h, volume = 4 ml/kg. The benefit of this schedule was to reduce the lethality of rotenone in a systemic model of PD (Teema et al., 2016; Alzahrani et al., 2018).

*Groups 3 and 4 (Rotenone + MTF 100 or 200 mg/kg):* Simultaneously, mice were treated with s.c. injections of rotenone (1 mg/kg, every 48 ± 2 h, nine doses) and oral MTF (100 or 200 mg/kg, every 24 ± 2 h, volume = 4 ml/kg).

*Groups 5 and 6 (Vehicle + MTF 100 or 200 mg/kg, respectively):* Mice were treated with s.c. injections of sunflower oil (4 ml/kg, every 48 ± 2 h, nine doses) and oral doses of MTF (100 or 200 mg/kg, every 24 ± 2 h, volume = 4 ml/kg). The results related to these groups are shown in the Supplementary Material (Supplementary Figures S1, S2).

Metformin was given by the aid of a gastric gavage tube and was continued until day 18. MTF was given on a daily basis at 8:00 h. The rotenone group received distilled water (4 ml/kg, p.o.) daily parallel to doses of MTF given in groups 3 and 4. The time course of the study is illustrated in Figure 1.

**FIGURE 1:** A scheme describing the study design.

### Assessment of the Motor Function of Mice

One day after the end of the therapeutic period (day 18), screening of mice motor functionality was achieved using the pole and rotarod tests.

#### Pole Test

Screening for the basal ganglia function is usually carried out by this test. A 50-cm-long pole of wood was put in the home cage at an inclined angle of about 40° on the room wall. To launch the test, mice were placed at the upper end of the pole with their faces upward, and then they reversed their body to face their home cage (time to turn) and climbed downward along the pole to arrive at the cage (time to descend) (Ogawa et al., 1985; Fleming et al., 2004). The two intervals were recorded (in seconds) using a stopwatch and compared for the study groups.

#### Rotarod Test

To monitor balance and motor coordination, each mouse was allocated individually on the rod (10 cm in length and 3 cm in diameter), the motor was turned on, and the speed was assessed at 18 rpm. Time spent from placement on the shaft of the rotarod until it falls to the ground (latency) was recorded, allowing each animal to remain on the rod for a maximum of 180 s (Zaitone et al., 2019).

### Processing of the Brains

Mice were euthanized under ketamine anesthesia (80 mg per kg, i.p.) (Gargiulo et al., 2012). Brains were dissected and rinsed with ice-cold phosphate-buffered saline (PBS, pH = 7.4). A brain hemisphere from each animal was rapidly frozen at −80°C for biochemical assays. Later, the striate were isolated from the frozen hemisphere, homogenized in PBS (10% w/v), and centrifuged and supernatants were harvested for biochemical assays while the second brain hemisphere was processed for preparing histologic slides. First, it was fixed in 4% paraformaldehyde solution overnight, and the midbrains were identified referring to a mouse brain atlas (Bregma −3.88 to −2.78) (Lein et al., 2007). After embedding in paraffin wax, two coronal sections (4 μm thick, first and third sections) were cut at the SN level (Zaitone et al., 2012b). Sections were deparaffinized and rehydrated for immunohistochemical staining as described later.

### Determination of Striatal Malondialdehyde, Reduced Glutathione, Hemoxygenase-1 Activity and Dopamine Level

Spectrophotometric measurement of reduced glutathione (GSH) and malondialdehyde (MDA) was done using kits obtained from Biodiagnostics (Cairo, Egypt). Using enzyme-linked immunosorbent assay (ELISA) kits, striatal levels of hemoxygenase-1 (mouse HO-1 ELISA kit, Abcam, catalog #ab204524) and dopamine (SunRedBio, Catalog #201-02-0668, Shanghai, China) were assayed. MDA, GSH, and dopamine levels were calculated as per gram of the striatal wet tissue weight; however, HO-1 activity was measured as pMol bilirubin/min/mg protein following the protocol described by the kit manufacturers. Results of the assays were read using a UV spectrophotometer (GSH and MDA) and an automated ELISA reader (HO-1 and dopamine) following the instructions of the manufacturer.

### Real-Time PCR Analysis of Nrf2, AMPK, FOXO3, and Thioredoxin

Striatal total RNA was extracted by the aid of an SV Total RNA Isolation System from Promega (WI, United States). RNA concentrations and purity were assessed by a NanoDrop ND-1000 spectrophotometer. Total RNA was transformed to cDNA using a SuperScript III First-Strand Synthesis System (#K1621, Fermentas, MA, United States). Gene expression was quantified via SYBR Green Master Mix (Applied Biosystems assay). Mouse-specific primers were forward (5′–3′) CGAGATATACGCAGGAGAGGTAAGA and reverse (5′–3′) GCTCGACAATGTTCTCCAGCTT for the nuclear factor erythroid 2–related factor 2 (Nrf2), forward (5′–3′) CCGCGGGAGACAAGCTT and reverse (5′–3′) GGAATGGAAGAAGGGCTTGATC for thioredoxin, forward (5′–3′) CTCAGTTCCTGGAGAAAGATGG and reverse (5′–3′) CTGCCGGTTGAGTATCTTCAC for AMPK α1, forward (5′–3′) TACGAGTGGATGGTGCGCTG and reverse (5′–3′) AGGTTGTGCCGGATGGAGTTC for FOXO3a, and forward CTGTGCAGGCTGCTGTAACG-3′ and reverse (5′-3)- AT GTAGGCCATGAGGTCCACC for β-actin. The PCR was carried by Applied Biosystem using software version 3.1 (StepOne^TM^). β-actin was used as a housekeeping gene for normalization. Gene expression was calculated using the comparative Ct method as previously described (Livak and Schmittgen, 2001), and the mRNA expression in each group was calculated relative to the value recorded in the vehicle control group.

### Western Blot Analysis of Nrf2, HO-1, AMPK, FOXO3, Thioredoxin, Cleaved Caspase 3, and VEGF

Total protein from the frozen striate was extracted by the aid of The ReadyPrep^TM^ protein extraction kit (Bio-Rad Inc., catalog #163-2086). Assessment of protein content was carried using the Bradford protein assay kit from Bio Basic Inc. (Markham Ontario L3R 8T4, Canada). Protein from each brain sample, 20 μg, was denaturized through boiling at 95°C for 5 min in buffer (4% SDS, 10% 2-mercaptoehtanol, 20% glycerol, 0.004% bromophenol blue, and 0.125 M Tris HCl, pH = 6.8). Then, protein was loaded in polyacrylamide gels that were relocated to a polyvinylidene difluoride (PVDF) membrane. After that, the PVDF membrane was blocked by tris-buffered saline with Tween 20 (TBST80) and 3% bovine serum albumin for 60 min at room temperature. PVDF membranes and primary mouse-specific antibodies of HO-1 (Abcam, catalog #ab13248), Nrf2 (Santa Cruz Biotechnology Inc., catalog #sc-365949), AMPK alpha-1 (Bioss Inc., catalog #bs-4002R), FOXO3 (MyBioSource, catalog #MBS151452), thioredoxin (Novus Biologicals, catalog #NB100-1634H), cleaved caspase 3 (c-caspase 3, Abcam, catalog #ab2302), and vascular endothelial growth factor (VEGF, Santa Cruz Biotechnology Inc., catalog #sc-7269), and β-actin (ThermoFisher, catalog #PA1-183) were incubated overnight at 4°C and rinsed (3–5 times/5 min) with TBST. Then, incubation was performed in horseradish peroxidase-conjugated secondary antibody (Goat anti-rabbit IgG antibody, Novus Biologicals) at room temperature for 60 min. The blot was rinsed with TBST80 and detected via chemiluminescent kit (Bio-Rad catalog #170-5060). Film bands were captured by a CCD camera-based imager (ImageQuantTMLAS500, GE Healthcare Life Sciences). Band intensity of the target proteins were quantified after normalization by β-actin using Image-J1.52p (National Institute of Health).

### Immunohistochemistry of Tyrosine Hydroxylase

Sections of 4 μm thickness were dried overnight at 37°C, then deparaffinized and rehydrated. Sections were stained using polyclonal rabbit tyrosine hydroxylase (TH) antibodies that were purchased from R&D systems. TH primary antibodies were diluted 1:800 with a primary antibody diluent (Genemed Biotechnologies, #10-001, CA) prior to use. Brain sections were incubated with the antibodies for 16 h at 4°C. Then, sections were washed and incubated with ready-to-use secondary antibodies for 20 min at room temperature. A Power-Stain^TM^ 1.0 poly HRP-3,3′-diaminobenzidine (DAB) kit was used to complete the staining process (Genemed Biotechnologies, catalog # 4-0017). Hematoxylin was used as a counterstain, rendering the stained structures visible under the microscope. Substantia nigra TH-positive neurons were evaluated using ImageJ software (NIH) according to previous methods (Cannon et al., 2009; Takeuchi et al., 2009). Briefly, the TH-stained sections were visualized, and the SNpc boundaries in the sections were defined and imaged at ×100 and ×400 magnification. Photomicrographs at ×100 magnification were taken by a PC-driven digital camera (Olympus E-620) fixed on Olympus CX31 light microscope (Tokyo, Japan). Then, images from the two immunostained sections were analyzed for the number of healthy TH-positive neurons characterized by visible nuclei and clear staining for TH. For counting the neurons, a blinded investigator utilized the ImageJ software, and the average of the neurons in the two sections/animal was taken and used in calculation.

### Statistical Analysis

Normally distributed data were presented as mean ± SD and statistically analyzed using Bonferroni’s *post hoc* test following a significant one-way ANOVA test. Non-parametric data belonging to the pole test were presented as median and quartile and statistically analyzed using Kruskal–Wallis ANOVA and Dunn’s *post hoc* test. *p* < 0.05 was the accepted level of significance. All possible comparisons were made among the study groups, and data were two-tailed.

## Results

### Motor Function Assessment

Assessment of mouse locomotor activity indicated significant prolongation in time (seconds) to turn and time to descend from the wooden pole to the home cage compared to the vehicle group (Figures 2A,B). MTF (200 mg/kg) prevented the loss of motor function induced by rotenone and led to shortening in these times (seconds). On the other hand, the time to turn and time to descend in mice treated with the vehicle + MTF 100 or 200 mg/kg was similar to that recorded in the vehicle group (Supplementary Figures S1A,B).

**FIGURE 2:** Effect of MTF on the locomotor activity of mice using **(A,B)** the pole test: presented as medians in boxplots, and analysis was done using the Kruskal–Wallis ANOVA and Dunn’s *post hoc* test with *P* < 0.05 as the accepted level of significance. **(C)** Rotarod test: results are expressed as mean ± SD and analyzed by applying one-way ANOVA followed by Bonferroni’s test with *p* < 0.05. #: Different from vehicle group, $: Different from rotenone group. *: Different from rotenone + MTF 100 mg/kg group at *p* < 0.05 (*n* = 6).

Similar locomotor dysfunction was observed in the rotarod test; the measured permanence time was shorter in the rotenone control group (20.14 ± 7.86) versus the vehicle group (178.71 ± 2.21, Figure 2C). MTF dose-dependently prolonged the permanence time for mice on the rod (54.14 ± 16.3 and 98.86 ± 18.87). Mice treated with the vehicle + MTF 100 or 200 mg/kg showed permanence times similar to that recorded in the vehicle group, and no significant difference was reported between them (179.17 ± 2.04 and 176.33 ± 5.99 versus 178.71 ± 2.21, Supplementary Figure S1C).

### Striatal Malondialdehyde, Reduced Glutathione, Hemoxygenase-1 and Dopamine

Figure 3 shows that the striatal level of MDA was greater, and GSH, dopamine, and HO-1 were decreased in the rotenone group versus the vehicle group (Figure 3). MTF (200 mg/kg) lessened MDA (Figure 3A) and enhanced GSH (Figure 3B) levels versus the rotenone control group. In addition, the higher dose of MTF prevented the loss of HO-1 and dopamine induced by rotenone (Figures 3C,D). Striatal dopamine level in groups 5 and 6 (mice treated with the vehicle + MTF, 100 or 200 mg/kg) was not significantly different from the level found in the vehicle group 1 (Supplementary Figure S2).

**FIGURE 3:** Effect of metformin on the striatal level of dopamine and oxidative stress markers in rotenone-parkinsonian mice. **(A)** MDA, **(B)** GSH, **(C)** HO-1, and **(D)** Dopamine. Results are expressed as mean ± SD and analyzed by applying one-way ANOVA followed by Bonferroni’s test. #: Different from vehicle group, $: Different from rotenone group. *: Different from rotenone + MTF 100 mg/kg group at *p* < 0.05 (*n* = 6).

### PCR Analysis for Nrf2, AMPK, FOXO3, and Thioredoxin

Measuring mRNA expression showed downregulation in genes encoding Nrf2 (∼25% of the control value, Figure 4A), thioredoxin (∼33% of the control value, Figure 4B), AMPK (∼50% of the control value, Figure 4C), and FOXO3 (∼60% of the control value, Figure 4D) in the rotenone control group versus the vehicle group. MTF dose-dependently upregulated the expression of Nrf2, thioredoxin, and AMPK. Both doses of MTF equally enhanced the expression of FOXO3 genes.

**FIGURE 4:** Effect of metformin on mRNA expression of AMPK and antioxidant markers in striata of rotenone-parkinsonian mice. Column charts for **(A)** Nrf2, **(B)** thioredoxin, **(C)** AMPK, and **(D)** FOXO3. mRNA expression in each group was calculated relative to the control value. Data are expressed as mean ± SD and analyzed using one-way ANOVA followed by Bonferroni’s test. #: Different from vehicle group, $: Different from rotenone group. *: Different from rotenone + MTF 100 mg/kg group at *p* < 0.05 (*n* = 6).

### Western Blot Analysis for Nrf2, HO-1, AMPK, FOXO3, and Thioredoxin

Nuclear factor erythroid 2–related factor 2, HO-1, AMPK, thioredoxin, and FOXO3 were decreased in the rotenone control group to significant levels. Treatment with MTF (100 and 200 mg/kg) diminished the effect of rotenone on these striatal parameters (Figures 5A,B–F). The effect of metformin on Nrf2, OH-1, and thioredoxin was dose-dependent.

**FIGURE 5:** Effect of metformin on striatal levels of proteins. **(A)** Western blotting of Nrf2, HO-1, AMPK, FOXO3, and thioredoxin versus β-actin was done using samples from brain striata. **(B–F)** Graphs present the densitometric analysis of western blotting of Nrf2, HO-1, AMPK, FOXO3, and thioredoxin, respectively. Data are mean ± SD for densitometric analysis of each gene relative to β-actin. Analysis was performed by applying one-way ANOVA followed by Bonferroni’s test #: Different from vehicle group, $: Different from rotenone group. *: Different from rotenone + MTF 100 mg/kg group at *p* < 0.05 (*n* = 3).

### Western Blot Analysis for Cleaved Caspase 3 and VEGF

On the other hand, Western blot results indicated greater c-caspase 3 and VEGF in the rotenone control group versus the vehicle group (∼3-fold and 2-fold increments, respectively, Figures 6A–C). Treatment with both doses of MTF produced a significant decrease in c-caspase 3 level, whereas MTF (200 mg/kg) was able to reduce VEGF significantly (Figures 6A–C).

**FIGURE 6:** Effect of metformin on striatal levels of c-caspase 3 and VEGF proteins. **(A)** Western blotting of c-caspase 3 and VEGF versus β-actin done using samples from brain striata. **(B,C)** Graphs present the densitometric analysis of western blotting of c-caspase 3 and VEGF. Data are mean ± SD for densitometric analysis of each gene relative to β-actin. Analysis was performed by applying one-way ANOVA followed by Bonferroni’s test. #: Different from vehicle group, $: Different from rotenone group. *: Different from rotenone + MTF 100 mg/kg group at *p* < 0.05 (*n* = 3).

### Immunohistochemistry for Tyrosine Hydroxylase

Tyrosine hydroxylase immunostaining revealed strong cytoplasmic staining in the vehicle control group in the SNpc region (Figure 7A, upper row). However, the rotenone control group showed reduced and irregular staining (Figure 7A). Images from the mice groups treated with MTF showed greater and regular area for staining (Figure 7A). Analyzing the number of TH-stained neurons showed the greatest number in the vehicle group, and this number was reduced significantly in the rotenone control group. Staining areas increased dose-dependently in mice receiving MTF (100 or 200 mg/kg) (Figure 7B). Similar results were obtained from striatal immunostaining; TH staining was strong and regular in the vehicle group (Figure 7A) but decreased and was sporadic in the rotenone control group (Figure 7A). Mice groups treated with MTF (100 or 200 mg/kg) showed gradual enhancement in staining (Figure 7A).

**FIGURE 7:** Immunohistochemistry staining for tyrosine hydroxylase in rotenone-parkinsonian mice. **(A)** The above panel shows images from the substantia nigra of the vehicle control group with multiple healthy TH-positive somas with regular shape and rounded large nuclei, and the striatum shows widespread positive regular staining. The image from the rotenone group shows a low number of healthy TH-positive cell somas and low scattered TH staining in the striatal nerve terminals. The rotenone + MTF 100 mg/kg group shows a higher number of TH-positive somas in the substantia nigra and higher striatal TH staining. The rotenone + MTF 200 mg/kg group shows improved TH staining in the cell somas and the striatal nerve terminals. **(B)** A column chart illustrating the number of TH-positive neurons per section in the substantia nigra pars compacta (left panel) and the striatal percent of TH-positive neurons (right panel). Results are expressed as mean ± SD and analyzed by applying one-way ANOVA followed by Bonferroni’s test. #: Different from vehicle group. $: Different from rotenone group. *: Different from rotenone + MTF 100 mg/kg group at *p* < 0.05 (*n* = 6).

Analysis of the striatal stained area indicated a significant decrease in the rotenone group versus the vehicle group (Figure 7B), and dose-dependent increments were observed in mice groups treated with MTF (Figure 7B). On the other hand, the mice in groups 5 and 6 treated with the vehicle + MTF 100 or 200 mg/kg showed intact SNpc neurons similar to those observed in the vehicle control group. Importantly, the number of the TH-positive neurons in groups 5 and 6 was not significantly different from that observed in the vehicle group (average ∼120 and ∼119 versus ∼124 neurons, Supplementary Figure S2).

## Discussion

The running work aims at exploring the antioxidant, antiangiogenic, and neuroprotective effect of MTF in a rotenone experimental model of PD. The work involved checking of the motor function, assessment of striatal biochemical oxidative stress, and angiogenesis and histopathological changes.

In the present study, mice injected with rotenone showed a significant dysfunction in initiation and coordination of locomotion. Furthermore, parkinsonian mice showed marked dopaminergic neurodegeneration in SNpc as expressed by lower TH-immunopositive neurons counted by image analysis software. Healthy TH-positive neurons in the SNpc of vehicle-treated mice were ∼124 neurons on average, and rotenone parkinsonian mice showed ∼29 neurons on average. Recently, Zhang et al. (2019) reported that the number of TH-positive neurons in the normal (contralateral) brain side was ∼59 cells and ∼28 cells in the damaged (ipsilateral) brain side in a 6-hydroxy-dopamine model of parkinsonism in mice. Although they obtained TH antibodies from a different source and used immunofluorescent staining, the results range was near to what was obtained in our study (Zhang et al., 2019). Meanwhile, other studies reported higher ranges for the number of TH-positive neurons when they used stereological analysis (Kaidery et al., 2013; Ahuja et al., 2016; Ismaiel et al., 2016; Katila et al., 2017; García-Domínguez et al., 2018). Thus, we can conclude that the three-dimensional maneuver in stereological analysis may give more accurate counting of cells, and this may explain the differences in the range of counted neurons.

In accordance with our findings, rotenone-treated animals showed motor abnormalities in the open field test associated with a manifest reduction in dopamine level (Zaitone et al., 2012a, b). Similar to our data, some studies reported dopamine level as ng/g of striatal wet tissues, and others represented it as ng/mg protein. The range of the measured dopamine in the experimental groups was 53.33–182.5 ng/g of striatal tissues. Consistently, Ho et al. (2019) used HPLC for detecting striatal dopamine and reported approximately 600 ng/g in normal mice. Another study highlighted that readings for the ELISA dopamine assay was in pg/ml; however, they did not mention the homogenization percentage, so it is not clear how much is the final concentration (Kim et al., 2019). Additionally, some studies reported dopamine level as ng/g of wet tissues, and others represented it as ng/mg protein.

Nevertheless, studies using HPLC analysis showed striatal dopamine levels higher than the data presented herein, which may be attributable to the higher sensitivity of the method. Discrepancy of the reported levels is present with a detection range from 650 to 100,000 ng/g as reported in several studies (Kaidery et al., 2013; Ahuja et al., 2016; Ismaiel et al., 2016; Katila et al., 2017; García-Domínguez et al., 2018; Ho et al., 2019).

In line with our data, many studies highlighted that rotenone-treated mice evoked poor mobility (Sindhu et al., 2005), nigrostriatal neurons loss (Betarbet et al., 2002), and striatal dopamine depletion (Alam and Schmidt, 2002).

Rotenone is an herbal extracted insecticide and an inhibitor of mitochondrial complex I. Some studies used systemic rotenone (1.5–2.5 mg/kg) to induce PD in experimental animals (Betarbet et al., 2000). In the current work, a new schedule for rotenone administration (1 mg/kg/s.c 48 h, nine doses) was applied; this schedule produces a systemic PD model without significant mortality.

The data presented herein reports an elevation in striatal MDA along with a reduction in GSH, Nrf2, and HO-1 expression in rotenone parkinsonian mice compared to vehicle-treated mice. Further, rotenone increased the striatal level of the angiogenesis marker, VEGF, and the apoptosis marker, c-caspase-3.

In line with our data, other researchers reported a reduction in SNpc GSH in PD postmortem brain tissues (Pearce et al., 1997) and elevated lipid peroxidation end products (Jenner, 2003). Furthermore, a recent meta-analysis on the quantification of blood oxidant stress indicators in patients with PD reported high blood MDA, 8-OH-deoxyguanosine, and ferritin as well as low glutathione, catalase, and uric acid (Wei et al., 2018).

The GSH level in parkinsonian mice may be attributable to Nrf2 deficiency. Nrf2 is a sensor and rectifier of cellular unbalanced redox states. Under oxidant stress, Nrf2 undertakes nuclear translocation from the cytoplasm to induce transcription of antioxidants. Nevertheless, this vital cellular defense mechanism is halted by inflammatory mediators and, consequently, Nrf2-induced glutathione-mediated cell survival (Hennig et al., 2018). Nrf2 nuclear localization in PD was observed, and the abundant oxidative stress outweighs Nrf2 capacity to prevent neuronal degeneration (Ramsey et al., 2007). Nrf2 enhances the expression of cellular antioxidant defenses, such as glutamate cysteine ligase, which catalyzes *de novo* synthesis of GSH (Kugiyama et al., 1998; Kansanen et al., 2013), HO-1 (Barakat et al., 2018), and thioredoxin (Ashino et al., 2013). Therefore, downregulation of Nrf2 expression was accompanied by lower HO-1 and thioredoxin expression according to the current study findings. In neuronal tissue, HO-1 is antioxidant protein upregulated in cellular oxidant stress (Nitti et al., 2018). Upregulation of HO-1 transcription is a downstream target of Nrf2 (Ishii et al., 2000). Cellular oxidant damage is associated with upregulation of HO-1, which enhances cell levels of bilirubin with antioxidant and radical scavenging properties (Nitti et al., 2018). In PD, HO-1 is reported to play a neuroprotective role (Hung et al., 2008; Song et al., 2009), and one study highlighted a pathogenic role for HO-1 in late stages of PD (Di Monte et al., 1995).

The current data displayed downregulation of striatal AMPK, FOXO3, and thioredoxin expression in rotenone parkinsonian mice in comparison to the vehicle group. In agreement, a previous study reported lower mitochondrial function, energy metabolic homeostasis, and AMPK function in PD following aging (Reznick et al., 2007). Indeed, neuronal bioenergetic failure increases their damage vulnerability (Goldberg et al., 2012). Diminished FOXO3 and thioredoxin expression may be related to the deficient AMPK-FOXO3 axis that upregulates thioredoxin expression (Li et al., 2009). Consistently, lower brain thioredoxin expression was reported in MPTP intoxicated mice (Kojima et al., 1999). Hence, the current situation includes reduced striatal GSH level, thioredoxin, and FOXO3 expression, highlighting that loss in Nrf2 and AMPK response favors dopaminergic neurodegeneration and motor alterations.

The data presented herein highlighted that MTF (100 or 200 mg/kg) prevented rotenone-induced motor dysfunction in the rotarod and pole tests and alleviated dopaminergic neurodegeneration. In agreement, MTF was reported to alleviate dopaminergic and mitochondrial dysfunction in the PD model in *drosophila* (Ng et al., 2012).

For confirming that the current doses of MTF did not produce a *per se* deleterious effect on the striatal neurons, the vehicle + MTF (100 and 200 mg/kg) groups were evaluated for motor function, striatal dopamine level, and SNpc TH-positive neurons. The results of these tests did not show changes in the studied markers compared to the vehicle control group, and this eliminates any harmful effects for MTF in the current doses and durations.

The current research showed the neuroprotective properties of MTF through antioxidant effects presented as a lower MDA level along with higher glutathione, Nrf2, HO-1, AMPK, FOXO3, and thioredoxin expression in MTF-treated mice compared to rotenone parkinsonian mice. Actually, MTF activates AMPK via elevating the AMP to ATP ratio or by initiating upstream regulators AMPK (Rena et al., 2017). Importantly, neuroprotective properties of MTF are mainly based on AMPK activation that may upregulate antioxidant capacity in three ways. First, AMPK enhances nuclear dislocation and accumulation of Nrf2, which upregulates antioxidant gene expression (Guerrero-Beltran et al., 2012; Joo et al., 2016). MTF pretreatment was documented to upregulate hippocampal Nrf2, HO-1, glutathione levels, and catalase activities of ischemic rats through AMPK activation (Ashabi et al., 2015). Moreover, Nrf2 overexpression attenuates neuronal mitochondrial complex II suppression regulating mitochondrial function (Esteras et al., 2016). Second, AMPK mediates GSH recycling via elevating NADPH produced from a pentose phosphate shunt (Jeon et al., 2012; Anandhan et al., 2017). Third, an *in vitro* study in human aortic endothelial cells displayed the role of MTF in reducing production of ROS from palmitic acid by increasing antioxidant thioredoxin through the AMPK-FOXO3 axis (Hou et al., 2010). Additionally, AMPK activated peroxisome proliferator-activated receptor-γ coactivator 1-α (PGC-1α) and FOXO3 implicated in glutathione peroxidase, catalase, superoxide dismutase, and uncoupling protein 2 transcription (Klotz et al., 2015; Jeon, 2016). Further, AMPK enhances FOXO3 implicated in transcription of proteins mediated autophagy and cell survival (Rosso et al., 2016). Hence, FOXO3 is considered as a pivotal transcription factor in detoxifying ROS and defending cells against oxidative stress.

The current study showed an elevated expression of the apoptotic marker, c-caspase 3, in the parkinsonian mice as compared to the normal vehicle-treated group. Similarly, c-caspase 3 immunostaining of postmortem brain of PD patients was found significantly higher than normal brains (Hartmann et al., 2000). Additionally, transgenic mice with disruption of the caspase-3 gene show endurance to MPTP-induced PD (Yamada et al., 2010). The current MTF-treated parkinsonian mice had significantly lower c-caspase 3 content as compared to rotenone-treated animals.

The data presented herein highlighted that rotenone increased the striatal VEGF level indicating enhanced angiogenesis. In PD, activated microglia cells release inflammatory and pro-angiogenic mediators (Antonella and Fabio, 2005). VEGF and vessel density were reported to increase in the SN of parkinsonian patients (Faucheux et al., 1999; Wada et al., 2006; Yasuda et al., 2007). Similar results were obtained from the SN of parkinsonian non-human primates, with which an increased number of VEGF-expressing neurons and an increment in the count of blood vessels were found (Barcia et al., 2005). Taken together, these observations propose that pathologic angiogenesis may accompany PD progression. The brain’s immature vessels lack the full blood–brain barrier characteristics, and hence, they allow peripheral molecules and immune cells to pass to brain parenchyma participating in the ongoing inflammatory cascade (Carvey et al., 2005).

The antiangiogenic effect of MTF is reported in many studies, including cancer (Zaafar et al., 2014; Orecchioni et al., 2015; Wang et al., 2015; Yang et al., 2017), stroke, and neurovascular disorders (Jin et al., 2014; Liu et al., 2014; Han et al., 2018). VEGF represents a major angiogenic marker that facilitates neovascularization with structural incompetency allowing for CNS trafficking of circulatory toxicants as well as inflammatory mediators. In the current work, an MTF neuroprotective effect through an antiangiogenic role has been elucidated. MTF-treated PD mice showed downregulation of VEGF expression when compared with untreated parkinsonian animals. VEGF upregulation can be attributed to the reduced neuronal GSH buffer as has been reported previously (Bir et al., 2013). Furthermore, dopaminergic neurons under oxidative stress exhibit an apoptotic tendency involving activated caspase-3, which enhances cellular survival defenses, including the angiogenic factors, such as VEGF.

Literature debated the neuronal protective effect of MTF. Animal studies reported the beneficial effect of MTF in murine models of PD through an AMPK energy equilibrating pathway (Patil et al., 2014), macroautophagic activation (Labuzek et al., 2010a; Lu et al., 2016; Katila et al., 2017), antioxidant (Patil et al., 2014; Lu et al., 2016), and anti-inflammatory actions (Labuzek et al., 2010b; Bayliss et al., 2016). Apparently, MTF treatment duration and dosage played a role in the MTF neuronal action. In their studies, de Pablos and colleagues have used a week therapy with MTF (150 mg/kg, p.o., twice daily dosage) in an MPTP-induced PD model and a model of dementia and showed a neuronal harming action of MTF. Hence, a warning conclusion was released for the possibility of the pathogenic role of MTF in neurodegenerative conditions (Ismaiel et al., 2016; Tayara et al., 2018). Based on the data reported by Patil et al. (2014), the neuroprotective role of MTF (500 mg/kg, p.o.) was not detected on the fifth day of therapy although it was significantly spotted in the 20th day and manifested as improved animal locomotive activity. Furthermore, the age of mice is another factor that may influence the utility of MTF; Thangthaeng et al. (2017) reported that MTF had no beneficial effects on aged mice (4 months old), and declines in spatial memory and visual acuity were observed in MTF treated groups. However, in the current study, 8- to 10-week-old mice were used, and favorable effects were obtained.

On the other hand, clinical studies were discouraging of the MTF neuroprotective role if used solo (Wahlqvist et al., 2012). Studies highlighted a higher risk of PD occurrence in long-term MTF treatment of over 50 diabetic patients compared to untreated controls (Kuan et al., 2017). This cannot be considered as a conclusive argument against the neuroprotective role of MTF. PD is a disease with a multifactorial pathogenesis, including environmental, genetic, and senescence variants. In clinical situations, the multivariate pathogenesis is represented, and in chemical models of PD using MPTP and rotenone, the main pathology is the deranged complex I energetic homeostasis. Curry et al. (2018), discussed the controversy of the MTF neuroprotective role and concluded that MTF may be of deleterious effect in early stages of PD although it is expected to be of clinical benefit in the advanced disease stages. Others attributed the possibility of MTF’s deleterious role in PD through hypovitaminosis B12 and called for further clinical studies paying attention to vitamin B12 monitoring during MTF therapy (Kuan et al., 2017).

## Conclusion

The running work shed light on the MTF neuroprotective properties via antiangiogenic, antioxidant, and anti-inflammatory activities. MTF upregulated AMPK-FOXO3 and thioredoxin proteins and downregulated striatal VEGF level. Accordingly, MTF can be considered as a promising drug in protection against PD progression in middle age, which requires further studies to establish its clinical validity.

## Data Availability Statement

All datasets generated for this study are included in the article/Supplementary Material.

## Ethics Statement

Experimental protocols and animal handling procedures were officially agreed by the Research Ethics Committee (Approval Number 201608RA4), Faculty of Pharmacy, Suez Canal University, in comply with the National Institute of Health Guide for the Care and Use of Laboratory Animals (NIH Publication No. 8023, revised 1978).

## Author Contributions

SHE and SYA received the fund for this project. SHE, HIB, ATI, DG, SYA, and SAZ conceived and designed the research. SHE, HIB, NEF, and SAZ conducted the animal experiments and analyzed the data. HIB contributed to biochemical assays. ATI and DG contributed to dhistopathological studies. All authors contributed to reagents or analytical tools, wrote, read, and approved the manuscript.

## Conflict of Interest

The authors declare that the research was conducted in the absence of any commercial or financial relationships that could be construed as a potential conflict of interest.
